This article has been retracted.

# MiR-744 increases tumorigenicity of pancreatic cancer by activating Wnt/β-catenin pathway

**DOI:** 10.18632/oncotarget.5317

**Published:** 2015-10-15

**Authors:** Wei Zhou, Yongfeng Li, Shanmiao Gou, Jiongxin Xiong, Heshui Wu, Chunyou Wang, Haijiao Yan, Tao Liu

**Affiliations:** ^1^ Pancreatic Disease Institute, Union Hospital, Tongji Medical College, Huazhong University of Science and Technology, Wuhan, Hubei, 430022, P.R. China; ^2^ Department of Oncology, the Third Affiliated Hospital of Soochow University, Changzhou, 213003, P.R. China; ^3^ Department of Digestive Surgical Oncology, Union Hospital, Tongji Medical College, Huazhong University of Science and Technology, Wuhan, Hubei, 430022, P.R. China

**Keywords:** miR-744, pancreatic cancer, Wnt/β-catenin signaling, cancer stem cells, tumorigenicity

## Abstract

The Wnt/β-catenin signaling pathway, commonly hyperactivated in pancreatic cancer, has been reported to play an important role in the maintenance of stemness of cancer stem cells (CSCs), which is closely related to the progression of pancreatic cancer. Therefore, exploring the regulatory mechanism in Wnt/β-catenin signaling may provide valuable clinical targets for cancer therapy. In the current study, we demonstrated that upregulation of miR-744 in pancreatic cancer promoted Wnt/β-catenin signaling by directly targeting secreted frizzled-related protein 1 (SFRP1), glycogen synthase kinase 3β (GSK3β), and transducin-like enhancer of split 3 (TLE3), important negative modulators of Wnt/β-catenin signaling. Expression of miR-744 was markedly upregulated in pancreatic cancer and positively correlated with poor patient survival. Furthermore, we found that overexpressing miR-744 enhanced, while inhibiting miR-744 reduced, the stem cell-like phenotype of pancreatic cancer cells *in vitro*. Importantly, *in vivo* model of human-derived pancreatic xenografts showed that miR-744 upregulation enhanced the tumorigenicity of pancreatic cancer cells. These findings suggest that miR-744 plays a vital role in promoting the stem cell-like phenotype of pancreatic cancer cells, and may represent a novel prognostic biomarker and therapeutic target.

## INTRODUCTION

Pancreatic cancer is one of the most aggressive and lethal malignancies and ranks as the eighth most frequent cause of cancer death worldwide [1, 2]. Despite the wide application of surgical resection and systemic chemo-radiotherapy, the overall 5-year survival rate for pancreatic cancer still remains between 3–5% and the median survival is less than 6 months [3–5]. Cancer stem cells (CSCs), a minor cohort of tumor cells with the ability to self-renew and generate the heterogeneous lineages of cancer cells, have been reported to play vital roles in tumor initiation and metastasis in numerous types of cancers [6, 7]. Similar, in pancreatic cancer, CSCs account for 0.2–0.8% of cancer cells and are reported to be essential for tumor growth, invasion, metastasis and recurrence [8–10]. However, the regulatory mechanism of CSCs in pancreatic cancer still remains largely unknown.

Aberrantly activated Wnt/β-catenin signaling pathway, contributes to the development and progression of multiple cancers, has been demonstrated as one of the most crucial pathways related with CSCs [11–13]. Activation of the Wnt/β-catenin signaling pathway in CSCs is responsible for their resistance to conventional therapies [14–16]. Additionally, hyper-activation of Wnt/β-catenin signaling has been showed to enhance stem cell–like phenotype of pancreatic cancer [17]. In the canonical Wnt pathway, ligand-receptor binding triggers the signaling cascade and releases β-catenin from the “destruction complex”, including Axin, adenomatous polyposis coli (APC), casein kinase 1α (CK1α), and glycogen synthase kinase 3β (GSK3β), resulting in nucleus translocation and interaction of β-catenin with TCF/LEF transcription factors and activating downstream target genes [18, 19].

On the other hand, it is well recognized that Wnt/β-catenin signaling is subject to multiple levels of negative control [20, 21]. In the absence of the Wnt signal, β-catenin could be degradated via ubiquitin-proteasome mechanism [22]. Another layer of regulation for suppression of β-catenin signaling is through secretion of antagonists of the Wnt pathway, such as secreted Frizzled-related proteins (SFRPs), Wnt inhibitory factor-1 (WIF1), and Dickkopf1 (DKK1) [23, 24]. Moreover, nuclear transcriptional suppressors including transducin-like enhancer of split 3 (TLE3) inhibit the transcriptional activity of LEF/TCF [25]. Thus, understanding how these negative regulatory effects on the Wnt/β-catenin signaling pathway are concomitantly deregulated in pancreatic cancer would be important for development of novel cancer treatment.

MicroRNAs (miRNAs) are endogenous non-coding small RNAs (17–25 nucleotides) that modulate gene expression at the post-transcriptional level [26]. Numerous miRNAs have been reported to maintain stemness and promote tumorigenicity of CSCs [27–29]. In the present study, we found that microRNA miR-744 was significantly upregulated in pancreatic cancer and enhanced a stem cell-like phenotype by inhibition of multiple negative regulators of Wnt/β-catenin pathway, including frizzled-related protein 1 (SFRP1), GSK3β, and TLE3. Therefore, our results suggest that deregulation of miR-744 may play an important role in maintenance of CSCs stemness and progression of pancreatic cancer.

## RESULTS

### MiR-744 overexpression correlates with pancreatic cancer progression

In order to investigate the important role of miRNA in pancreatic cancer, published miRNA expression profiles consisting of 136 pancreatic cancer tissues and 22 normal pancreatic tissues (NCBI/GEO/GSE24279) was analyzed. We found that miR-744 was significantly upregulated in tumor tissues compared to normal tissues (Fig. 1A). Consistently, real-time PCR analysis revealed that miR-744 was ubiquitously overexpressed in 8 pancreatic cancer cell lines compared with two HPDECs, and in 8 pancreatic cancer samples compared with two normal pancreatic tissues (Fig. 1B–1C). Collectively, these findings suggest that miR-744 expression is increased in pancreatic cancer.

**Figure 1:** MiR-744 overexpression positively correlates with pancreatic cancer progression **A.** Expression profiling of miR-744 from published microarray-based high-throughput datasets (*n* = 158; NCBI/GEO/GSE24279). **B.** RT- PCR analysis of miR-744 expression in 8 pancreatic cancer cell lines and 2 HPDECs. Transcript levels were normalized to *U6* expression. Each bar represents the mean ± SD of three independent experiments. *P < 0.05. **C.** RT- PCR analysis of miR-744 expression in 8 pancreatic cancer samples and 2 normal pancreatic tissues. **D.** miR-744 expression was positively correlated with clinical stages of pancreatic cancer. **E–F.** Overall survival **E.** and disease-free survival **F.** of pancreatic cancer patients with low- versus high-expression of miR-744 (*n* = 80; *P* < 0.05).

The clinical relevance of miR-744 in pancreatic cancer progression was further investigated in a cohort of 80 archived human pancreatic cancer specimens (Supplementary Table 1). Statistical analysis revealed that miR-744 expression was positively correlated with clinical stage in patients with pancreatic cancer (*P* < 0.05) (Fig. 1D and Supplementary Table 1). Importantly, patients with higher miR-744 expression had a shorter survival time, whereas patients with lower miR-744 expression showed a longer survival time and disease-free survival (*P* < 0.05; *P* < 0.05; Fig. 1E–1F). Moreover, univariate and multivariate analyses indicated that miR-744 expression and clinical stage are independent prognostic factors in pancreatic cancer (Supplementary Table 2). Taken together, these results indicate a possible link between miR-744 overexpression and human pancreatic cancer progression.

### Upregulation of miR-744 promotes CSC-like traits in pancreatic cancer cells

To understand the biological role of miR-744 in pancreatic cancer progression, miR-744 was stably transduced into the MIA PaCa-2 and AsPC-1 pancreatic cancer cell lines via retroviral- and lentiviral-vector to generate MIA PaCa-2/miR-744 and AsPC-1/miR-744 cell lines (Supplemental Fig. 1A). A tumor sphere formation assay showed that miR-744-transduced cells formed a larger number of spheres with increased diameter compared to vector control cells (Fig. 2A–2B and Supplemental Fig. 1B). Additionally, populations of cells that were positive for the pancreatic CSC marker CD133 and SP positive cells were dramatically increased in miR-744-transduced cells compared with vector control cells (Fig. 2C–2D). Furthermore, we found that miR-744 overexpression significantly upregulated the mRNA expression levels of multiple pluripotency factors, including BMI1, ABCG2, OCT4, SOX2, and NANOG (Fig. 2E). Collectively, our results suggest that miR-744 overexpression promotes a stem cell-like phenotype in pancreatic cancer cells.

**Figure 2:** MiR-744 overexpression promotes pancreatic cancer stem cell-like traits **A–B.** Representative micrographs A. and quantification B. of tumorsphere formation in pMSCV-miR-744-overexpressing cells or pMSCV-vector cells. Scale bar, 100 μm. **C.** Hoechst 33342 dye exclusion assay showing the effect of pMSCV-miR-744-overexpressing cells or pMSCV-vector cells on side population cells. **D.** Distribution of CD133^+^ cells using flow cytometric analysis. **E.** qRT-PCR analysis of mRNA expression of stem cell markers in the indicated cells. Transcript levels were normalized to GAPDH expression. Error bars represent mean ± SD from three independent experiments. *P < 0.05

### Inhibition of miR-744 suppresses a CSC-like phenotype in pancreatic cancer cells

Silencing endogenous miR-744 using antagomir-744, an antisense-based specific inhibitor against miR-744, dramatically inhibited the capability of tumor sphere formation in both MIA PaCa-2 and AsPC-1 pancreatic cancer cells (Supplemental Fig. 2A and Fig. 3A–3B). Furthermore, we found that miR-744 inhibition significantly reduced the populations of CD133^+^ and SP^+^ cell and decreased mRNA expression of BMI1, ABCG2, OCT4, SOX2, and NANOG (Fig. 3C–3E). Thus, our experiments further indicate that miR-744 might act as a CSC inducer.

**Figure 3:** MiR-744 inhibition suppresses pancreatic cancer stem cell-like phenotype **A–B.** Representative micrographs A. and quantification B. of tumorsphere formation in antagomir-744 or control cells. Scale bar, 100 μm. **C.** Effects of antagomir-744 or control cells on side population cells. **D.** Distribution of CD133^+^ cells using flow cytometric analysis. **E.** qRT-PCR analysis of mRNA expression of pluripotency-associated markers in antagomir-744 or control cells. Transcript levels were normalized to *GAPDH* expression. Error bars represent mean ± SD from three independent experiments. *P < 0.05.

### Upregulation of miR-744 promotes tumorigenicity of pancreatic cancer cells *in vivo*

The biological effect of miR-744 on pancreatic cancer progression was further examined using an *in vivo* tumor model. MIA PaCa-2/miR-744 or MIA PaCa-2/vector cells were subcutaneously xenografted into NOD/SCID mice. As shown in Fig. 4A–4D and Supplemental Fig. 3A–3B, the tumors formed by MIA PaCa-2/miR-744 cells were larger in size and had increased weight, compared with the tumors formed from the vector control cells. In contrast, when endogenous miR-744 was inhibited using miRZip744, the tumors were smaller in size and had decreased weight than those formed by control cells (Fig. 4A–4C). The tumors formed by MIA PaCa-2/miR-744 cells were significantly larger than the vector control tumors, when 1 × 10^5^ or 1 × 10^4^ cells mixed with matrigel were subcutaneously inoculated into the mice. Importantly, only MIA PaCa-2/miR-744 cells formed tumors when 1 × 10^3^ cells were implanted (Fig. 4D). These results indicate that miR-744 promotes pancreatic cancer tumorigenicity *in vivo*.

**Figure 4:** Upregulation of miR-744 promotes tumorigenicity of pancreatic cancer cells *in vivo* **A.** Tumors formed by MIA PaCa-2/pMSCV-miR-744 cells in a nude mouse xenograft model were larger in diameter than vector control tumors in the 1 × 10^5^ cells group. Conversely, tumors formed by MIA PaCa-2/miRZip-744 cells were smaller than tumors formed by control cells. Only miR-744-overexpressing cells formed tumors following implantation of 1 × 10^3^ cells. Representative images of the tumors are shown. **B.** Histograms depicting the mean tumor weights of each group (*n* = 5 per group). *P < 0.05. **C.** Growth curves for tumor formation after implantation. Mean tumor volumes are plotted. **D.** Tumor formation initiated by the indicated cells in BALB/C nude mice.

### MiR-744 activates Wnt/β-catenin pathway by targeting SFRP1, GSK3β, and TLE3

Using publicly available algorithms (TargetScan6.2 and miRanda), we found that SFRP1, GSK3β, and TLE3, negative regulators of the Wnt/β-catenin pathway, might be the potential targets of miR-744 (Fig. 5A). Western blot analysis revealed that the expression of SFRP1, GSK3β and TLE3 was markedly decreased in miR-744-transduced cells but elevated in antagomir-744-transfected cells (Fig. 5B). However, neither miR-744 overexpression nor miR-744 inhibition has effect on the mRNA levels of SFRP1, GSK3β, and TLE3, suggesting that the inhibitory effect of miR-744 on SFRP1, GSK3β, and TLE3 was regulated at the post-transcriptional level (Supplemental Fig. 4A). In addition, the results of the luciferase reporter assay indicated that miR-744 overexpression significantly repressed, whereas inhibition of endogenous miR-744 increased, the luciferase activity of 3′UTRs of SFRP1, GSK3β, and TLE3, while ectopically expressing mutant miR-744 had no inhibitory effect on the 3′UTRs luciferase activity (Fig. 5C). Importantly, results of the miRNP immunoprecipitation assay showed that miR-744 selectively associated with SFRP1, GSK3β and TLE3 (Fig. 5D), further demonstrating that SFRP1, GSK3β, and TLE3 are targets of miR-744.

**Figure 5:** MiR-744 directly targets SFRP1, GSK3β and TLE3 **A.** Predicted miR-744 target sequences in the 3′-UTRs of SFRP1, GSK3β, TLE3 and a mutant containing three altered nucleotides in the seed sequence of miR-744 (miR-744-mu). **B.** Western blot analysis of SFRP1, GSK3β, TLE3 and nuclear β-catenin in the indicated cells. α-Tubulin served as the loading control. **C.** Luciferase activity of target 3′UTR in the indicated cells. **D.** RIP as assessed by Ago2 IP. IgG immunoprecipitation was used as the negative control. **E.** The indicated cells transfected with TOP flash/FOP flash and Renilla pRL-TK plasmids were subjected to dual-luciferase assays 48 hours after transfection. Reporter activity detected was normalized by Renilla luciferase activity. **F.** Luciferase activity of TOP flash/FOP flash in the indicated cells. Each bar represents the mean ± SD of three independent experiments. *P < 0.05.

As expected, we found that miR-744 overexpression increased, while miR-744 inhibition reduced the luciferase activity of the TOP flash/ FOP flash reporter, and mutant miR-744 had no effect (Fig. 5E), indicating that miR-744 activates Wnt/β-catenin signaling. Silencing SFRP1, GSK3β and TLE3 disrupted the repression efficacy of the miR-744-regulated Wnt/ β-catenin activity (Supplemental Fig. 4B and Fig. 5F), suggesting that miR-744 activates Wnt/β-catenin signaling through suppressing SFRP1, GSK3β, and TLE3. Moreover, the expression of miR-744 and nuclear β-catenin was significantly increased in the tumors formed by miR-744-overexpressing cells but decreased in mR-744-inhibited tumors. Whereas, the levels of SFRP1, GSK3β and TLE3 dramatically decreased in the mice tumors formed by miR-744-overexpressing cells and increased in the mR-744-inhibited tumors (Supplemental Fig. 3A and 4C). In addition, tumor sphere formation showed that the inhibitive effect of downregulating miR-744 was antagonized by silencing of SFRP1, GSK3β, and TLE3 (Supplemental Fig. 4D). These results demonstrate that SFRP1, GSK3β and TLE3 are key regulators for miR-744 -induced Wnt/β-catenin activation and stem cell-like traits in pancreatic cancer cell lines.

### MiR-744 is clinically correlated with Wnt/β-catenin activation in pancreatic cancer

To further determine the clinical correlation between miR-744 and the Wnt/β-catenin signaling pathway, we examined whether miR-744–induced suppression of SFRP1, GSK3β, and TLE3 and β-catenin nuclear accumulation in pancreatic cancer are relevant in clinical samples. Using 8 freshly collected clinical pancreatic cancer samples, we found that miR-744 expression was inversely correlated with expression of β-catenin (*r* = 0.62, *P* < 0.05), SFRP1 (*r* = −0.89, *P* < 0.05), GSK3β (*r* = −0.61, *P* < 0.05), TLE3 (*r* = −0.82, *P* < 0.05) (Fig. 6A–6C). In consistent with previous reports [30, 31], tumor sphere formation assay revealed that CD133^+^ pancreatic cancer cells isolated from pancreatic cancer tissues formed more spheres than the CD133^−^ pancreatic cancer cells (Supplemental Fig. 5A). Furthermore, we found that the expression of miR-744 and nuclear β-catenin was significant higher in CD133^+^ pancreatic cancer cells higher than that in CD133^−^ pancreatic cancer cells. Whereas the levels of SFRP1, GSK3β and TLE3 in the CD133+ pancreatic cancer cells were dramatically lower compare with CD133^−^ pancreatic cancer cells (Supplemental Fig. 5B–5C), which further support the hypothesis that miR-744 upregulation activates the Wnt/β-catenin signaling via downregulation of SFRP1, GSK3β and TLE3 in pancreatic cancer.

**Figure 6:** MiR-744 is clinically correlated with nuclear β-catenin and expression of its targets in pancreatic cancer **A.** qRT-PCR of miR-744 expression in 8 fresh pancreatic cancer tissues and 2 normal pancreatic tissues. *U6* was used as the control for RNA loading; miRNA levels were normalized to miR-744 expression of sample one. Each bar represents the mean ± SD of three independent experiments. **B.** Western blot of SFRP1, GSK3β, TLE3 and nuclear β-catenin in 8 fresh pancreatic cancer tissues and 2 normal pancreatic tissues. α-Tubulin was used as the loading control. **C.** Correlation between miR-744 expression levels and SFRP1, GSK3β, TLE3 and nuclear β-catenin in pancreatic cancer clinical tissues. The expression levels of SFRP1, GSK3β, TLE3 and β-catenin, checked by western blotting analysis, were determined by densitometry. The ratio of first sample (SFRP1/α-tubulin, GSK3β/α-tubulin, TLE3/α-tubulin and nuclear β-catenin /α-tubulin) was considered as 1.0.

## DISCUSSION

Numerous studies have demonstrated that pancreatic CSCs are clinically correlated with cancer invasion, metastasis and chemo-resistance, which leads to high morbidity and mortality among patients [9, 32, 33]. However, the mechanism how pancreatic CSCs maintain a stem cell-like phenotype remains unclear. Herein, we found that the overexpression of miR-744 in pancreatic cancer enhanced, whereas suppression of miR-744 inhibited, the CSC-like phenotypes. Consistently, *in vivo* studies revealed that silencing mir-744 significantly inhibited the tumorigenicity of pancreatic cancer cells. These findings uncover a novel mechanism for pancreatic CSCs maintenance and suggest a potential therapeutic effect of miR-744.

Despite multiple layers of negative regulation, high activation of the Wnt/β-catenin signaling pathway has been observed in various types of cancers, including pancreatic cancer [34, 35]. How cancer cells override negative modulation and maintain hyper-activation of Wnt/β-catenin signaling is still unknown. Herein, we found that overexpression of miR-744 enhanced, while suppression of miR-744 inhibited Wnt/β-catenin signaling through directly targeting different levels of negative regulators of the pathway, including SFRP1, GSK3β and TLE3. Furthermore, nuclear β-catenin positively correlated, while SFRP1, GSK3β and TLE3 expression inversely correlated with the expression of miR-744 in pancreatic cancer clinical specimen. These findings suggest a novel mechanism in which Wnt/β-catenin signaling is constitutively activated in pancreatic cancers.

Dysregulation of SFRP1, GSK3β and TLE3, three important negative modulators of Wnt/β-catenin signaling, contribute to carcinogenesis [36, 37]. For instance, SFRP1 has been shown to inhibit epithelial-mesenchymal transition in A549 human lung adenocarcinoma cell line [38]. Delic S et al. reported that SFRP1 was downregulated in glioma cells and promoted cancer invasion [39]. SFRP1 has been demonstrated to act as a favorable prognostic factor in human biliary tract carcinoma [40]. GSK3β is found to be downregulated in various cancers that result in removal of the inhibitory effect of the Wnt/β-catenin signaling pathway [41, 42]. TLE3 expression is reported to be associated with sensitivity to taxane treatment in ovarian carcinoma [43]. In the current study, SFRP1, GSK3β and TLE3 were directly targeted and simultaneously downregulated by miR-744 in pancreatic cancer, and the expression of SFRP1, GSK3β and TLE3 was inversely correlated with the expression of miR-744 in pancreatic cancer tissues. These data suggest a novel regulatory mechanism for SFRP1, GSK3β and TLE3, and indicate that decreased expression of SFRP1, GSK3β and TLE3 could enhance cancer cell stemness.

Due to the significant impact upon cancer progression, anti-tumor drugs targeting Wnt/β-catenin have aroused great interest worldwide [44, 45]. Althorugh kinase inhibitors have become the preferable anti-tumor target for pharmaceutical synthesis [44], the two main kinases involved in the Wnt/β-catenin pathway, namely CK1a and GSK3β, negatively modulate signaling and cannot serve as therapeutic targets for anti-tumor treatment. Therefore, it is of urgent need to discover novel molecules that play vital roles in the regulation of the Wnt/β-catenin pathway [46, 47]. In the current study, we found that miR-744, an endogenous small RNA, markedly activated the Wnt/β-catenin signaling via inhibition of multiple negative regulators of the pathway, including GSK3β. Moreover, the expression of miR-744 was positively correlated with tumorgenesis both *in vitro* and *in vivo*. These findings suggest miR-744 as a potential therapeutic target.

Analysis of the miR-744 promoter region using the CONSITE program predicted two typical NF-κB-responsive elements and one typical TGF-β-responsive elements (SRE). Previously, it has been reported that tumor microenvironments, induced by NF-κB and TGF-β signaling, play important roles in progression and development of pancreatic cancer, such as proliferation, metastasis and cancer stem cell-like phenotype [33, 48–50]. Thus, it would be of great interest to further investigate whether upregulation of miR-744 in pancreatic cancer is attributed to NF-κB and/or TGF-β-mediated transcriptional upregulation.

In summary, this study demonstrated that overexpression of miR-744 promoted stem cell-like phenotype and tumorigenecity in pancreatic cancer cells by directly targeting multiple negative modulators of Wnt/β-catenin pathway, namely SFRP1, GSK3β and TLE3. These findings reveal a novel molecular mechanism on how aberrant activation of the Wnt/β-catenin pathway is maintained in cancer and suggests that miR-744 might serve as a potential therapeutic target for pancreatic cancer.

## MATERIALS AND METHODS

### Cells

The pancreatic cancer cell lines, including AsPC-1, Capan-1, Bxpc-3, CFPAC-1, Hs667T, Capan-2, MIA PaCa-2 and PANC-1were grown in the DMEM medium (Invitrogen, Carlsbad, CA) supplemented with 10% fetal bovine serum (HyClone, Logan, UT). Primary cultures of normal human pancreatic duct epithelial cells (HPDEC) were maintained in keratinocyte serum-free medium (KSFM; Gibco) with EGF (1 ng/ml) and BPE (50 mg/ml). All cells were incubated at 37°C in a humidified atmosphere with 5% CO2.

### Patient information and tissue specimens

A total of 80 paraffin-embedded and archived pancreatic cancer samples, which were histopathologically and clinically diagnosed at the Huazhong University of Science and Technology Union Hospital from 2001 to 2006, were examined in this study. The 8 freshly collected pancreatic cancer samples, including clinical stage I: 1, stage II: 3, stage III: 2 and stage IV: 2, were frozen and stored in liquid nitrogen until required. Prior patient consent and approval from the Institutional Research Ethics Committee were obtained for the use of these clinical materials for research purposes. Clinical information on the samples is summarized in Supplementary Table 1. Diagnosis was based on pathological evidence, and the specimens were immediately snap-frozen and stored in liquid nitrogen tanks. For the use of these clinical materials for research purposes, prior patients' consents and approval from the Institutional Research Ethics Committee were obtained.

### Vectors, retroviral infection and transfection

The human miR-744 gene was PCR-amplified from genomic DNA and cloned into a pMSCV-puro retroviral vector or pSin4-EF2-IRES-Puro lentiviral vector. The miR-744 anti-sense was cloned into miRZip plasmid purchased from System Biosciences and used according to previous report [51]. Antagomir-744 was purchased from RIBOBIO Company (Guangzhou, China). pMSCV-miR-744, pSin4-miR-744 or miRZip-744 were cotransfected with the pIK packaging plasmid in HEK293T cells using the standard calcium phosphate transfection method. Supernatants were collected after 36 cotransfection and incubated with cells for 24 hours in the presence of polybrene (2.5 μg/ml). After infection, puromycin (0.5 μg/ml) was used to select stably transduced cells over a 10-day period [52]. The reporter plasmids containing wild-type (CCTTTGATC; TOP flash) or mutated (CCTTTGGCC; FOP flash) TCF/LEF DNA binding sites were purchased from Upstate Biotechnology (New York, USA). The 3′UTRs of SFRP1, GSK3β and TLE3, respectively, were amplified and cloned downstream to the luciferase gene in a modified pGL3 control vector.

### Primers and Oligonucleotides

Cloning miR-744: 5′-GCCAGATCTTTTCACT GCAG AGGACTTGAAAGAC-3′ and 5′-GCCGAATTC AATAGGACACTAATAGGAAGATG AT -3′; Cloning sFRP1-3′UTR-luci: GCCCCGCGGCGCCTGTCAGTA GTGGACATTGTAA -3′ and 5′-GCCCTGCAG TCC ATAGGCAATCAAGTTCAAAGGA -3′; Cloning GSK3β- 3′UTR-luci: 5′-GCCCCGCGG TTTCACTCGCTG TTTAGC -3′ and 5′-GCCCTGCAG GGTCTATCAA CGCCACTA-3′; Cloning TLE3–3′UTR-luci: 5′-GCCCC GCGG GTTGGTTTGATTGTTGCGTCTT-3′and 5′-GC CCTGCAG TGCTGCG ATGCTGGGTAT-3′. For depletion of SFRP1, GSK3βand TLE3 siRNA was synthesized and purified by RIBOBIO Company (Guangzhou, China).

### Western blot analysis

Western blot analysis was performed using anti- SFRP1 (1:200); anti-GSK-3β antibody (1:500), anti-TLE3 (1:500), anti-β-catenin (1:500) antibodies (Abcam, Cambridge, MA, USA). To control sample loading, the blotting membranes were stripped and re-probed with an anti–α-tubulin antibody (1:1000, Sigma, Saint Louis, MO, USA). Nuclear extracts were prepared using the Nuclear Extraction Kit (Active Motif), according to the manufacturer's instructions. Briefly, cells were collected in the PBS/phosphatase inhibitors solution and lysed in the Lysis Buffer, and then centrifuged for 5 minutes. Suspending nuclear pellet in 50ul Complete Lysis Buffer, then incubating for 30 minutes on ice. Vortex the mixture for 30 seconds followed by centrifuge for 10 minutes at 14,000 g at 4°C, the collected nuclear extraction were store at −80°C for further examination. The expression levels of SFRP1, AXIN2, ICAT and β-catenin were determined by densitometry. The ratio of first sample (SFRP1/α-tubulin, AXIN2/α-tubulin, ICAT/α-tubulin and β-catenin /α-tubulin) was considered as 1.0.

### Tumor sphere formation assay

Five hundred cells were seeded in 6-well ultra-low cluster plates and 10 or 20 cells were seeded in 24-well ultra-low cluster plates for 10 days. Spheres were cultured in DMEM/F12 serum-free medium (Invitrogen, USA) supplemented with 2% B27 (Invitrogen, USA), 20 ng/ml EGF, 20 ng/ml bFGF, and 5 μg/ml insulin (PeproTech, USA).

### Flow cytometric analysis

Cells were dissociated with trypsin and suspended at 1 × 10^6^ cells/mL in DMEM containing 2% FBS, and then incubated at 37°C for 30 minutes with or without 100 μM verapamil (Sigma-Aldrich) to inhibit ATP-binding cassette (ABC) transporters. The cells were subsequently incubated for 90 minutes at 37°C with 5 μg/mL Hoechst 33342 (Sigma-Aldrich). Lastly, cells were incubated on ice for 10 minutes and washed with ice-cold phosphate-buffered saline (PBS) prior to flow cytometry analysis. Flow cytometric analysis or flow cytometric cell sorting was conducted using fluorescein isothiocyanate (FITC)-conjugated monocloncal mouse anti-human CD133 (Miltenyi Biotec GmbH, Germany). Samples were analyzed and sorted on BD FACSCanto II and FACSAria I, respectively (BD Biosciences, USA) with data analyzed using FlowJo software (Tree Star Inc, USA).

### Animal studies

All experimental procedures were approved by the Institutional Animal Care and Use Committee (IACUC) of Guiyang Medical College. The 6-week-old BALB/c-nu mice were randomly divided into three groups (*n* = 5 per group). Cells (1 × 10^5^, 1 × 10^4^, 1 × 10^3^) were inoculated subcutaneously together with Matrigel (final concentration of 25%) into the inguinal folds of the nude mice. Tumor volume was determined using an external caliper and calculated using the equation (L × W^2^)/2. The mice were sacrificed 35 days after inoculation and the tumors were excised and subjected to pathologic examination.

### Luciferase reporter assay

Cells were plated in 100-mm cell culture dishes, proliferating to 60–80% confluence after 24 h of culture. The reporter constructs were transfected using Lipofectamine 2000 (Life Technologies) according to the manufacturer's protocol. After 12-h incubation, the transfection medium was replaced, cells were harvested and washed with PBS (pH 7.4), and lysed with passive lysis buffer (Promega). The cell lysates were analyzed immediately using a 96-well plate luminometer (Berthold Detection System, Pforzheim, Germany). Luciferase and Renilla luciferase were measured using a Dual-Luciferase Reporter Assay System (Promega) according to the manufacturer's instructions. The luciferase activity of each lysate was normalized to Renilla luciferase activity. The relative transcriptional activity was converted into fold induction above the vehicle control value.

### Statistical analysis

All statistical analyses were carried out using SPSS 18.0 statistical software. The Kaplan-Meier method was used to establish survival curves, and the survival differences were compared using the log-rank test. Continuous data were compared using Student's 2-tailed *t*-test. Multivariate statistical analysis was performed using a Cox regression model. In all cases, *P* < 0.05 was considered statistically significant.

## SUPPLEMENTARY FIGURES AND TABLES


